RETRACTED

# Quantifying the Soil Arthropod Diversity in Urban Forest in Dera Ghazi Khan

**DOI:** 10.1155/2022/8125585

**Published:** 2022-09-22

**Authors:** Muhammad Mohsin, Haseeb Ahmad, Muhammad Nabeel Nasir, Zain Ul Abideen, Muhammad Nadeem, Rukhsana Sattar, Abdul Qadeer Saad, Mujahid Hussain, Syed Akbar Shah, Hanlie Cheng, David Sturdivant, Syeda Amber Hameed

**Affiliations:** ^1^Department of Zoology, Ghazi University Dera, Ghazi Khan, Pakistan; ^2^Rural Dispensary Chak No. 151JB, Tehsil Chiniot, District Chiniot, Pakistan; ^3^District Headquarter Hospital, Rajanpur, Pakistan; ^4^Department of Zoology, Cholistan University of Veterinary and Animal Sciences, Bahawalpur, Pakistan; ^5^School of Energy Resource, China University of Geosciences (Beijing), Beijing 434000, China; ^6^The King's School, BP1560, Bujumbura, Burundi

## Abstract

Arthropods can be either large or too small to be seen from the microscope. Their legs are jointed and perform a specific function in the soil. Several arthropods have been identified to date. Therefore, it is essential to identify them in a different type of soil. An experiment to quantify the soil arthropods in the urban forests of D.G. Khan was conducted at the Zoology lab of Ghazi University on four tree plants, i.e., neem (*Azadirachta indica*), mango (*Mangifera indica*), guava (*Psidium guajava*), and phalsa (*Grewia asiatica*). Soil samples were taken from different areas and on different months. The diversity of arthropods was analyzed through the Shannon index. The results were all significant. The total number of arthropods found in the experiment was 5151, with the following distributions: millipedes were 132 in neem, 133 in guava, 113 in mango, and 121 in phalsa; centipedes were 136 in neem, 142 in guava, 118 in mango, and 132 in phalsa; springtails were 138 in neem, 130 in guava, 120 in mango, and 134 in phalsa. There were a total of 12 different species of arthropods found. Neem (*Azadirachta indica)* have mites, centipede, and ants; guava (*Psidium guajava)* have centipedes and ants. Mango (*Mangifera indica)* have millipedes, centipedes, mites, springtail, and ants, and phalsa (*Grewia asiatica)* have mites, ants, and centipedes. The study reveals that millipedes, centipedes, springtails, and ants were found abundantly in the urban forest area of D.G. Khan, resulting in increased organic matter decomposition and appropriate distribution of nutrients through the soil having beneficial effects on the terrestrial ecosystem.

## 1. Introduction

Arthropods are soil invertebratess that can be large or quite microscopic, have jointed legs, and perform particular functions in the the soil community. Due to the body, widths can be classified into two forms mesofauna and macrofauna, also termed microarthropod (0.2 mm) and macroarthropod (2 mm). Arthropod includes the class of insect. The lightest insects weigh less than 25 micrograms; the heaviest, however, weigh more than 70 grams (2.5 oz) [1]. Few of their organisms have wingless like springtails and many have wings on their body. The most abundant soil arthropods are Acari (mites and collembolans) and springtail. Springtails have segmented body and wingless, ranging from 0.2 to 6 mm, with specialized appendages used for jumping. The most conspicuous segmental specialization is in the brain. For Symphypleona in the age maturity, most of them are soil dwellers range from 50 to 100,000 individuals m^−2^. Some different species of collembolan like Protura and diploma are also wingless insects. In 1992, a take look anticipated that in Costa Rica alone, there were 500,000 species of animals and plants, of which 365,000 had been arthropods [2].

RETRACTED

Some other species act as predators in nature, feeding on small fauna. And few have scavengers. Soil arthropods are microscopic or big period invertebrates with jointed legs. They play big roles within the soil network. Based on body width, soil arthropods may be labeled mesofauna and macrofauna. They can be categorized additionally as microarthropods (0.2–2 mm) or macroarthropods (>2 mm). According to standard taxonomy, soil arthropods fall underneath beauty insects (e.g., Protura, Diplura, Collembola, and big insects); class Myriapoda (Symphyla and Pauropoda), class Crustacean (Tardigrada, Copepods and Isopoda), and sophistication Arachnidan (Pseudoscorpiones, Arana, and Acari). Acari (mites) and collembolans (springtails) are the most sizable soil microarthropods in terms of the range of individuals and species [3]. Springtails are wingless bugs with the segmented bodies (0.2–6 mm) and specialized appendages, in addition to a spring-like tail for jumping. Most species are dwellers of soil or litter, while few live on the floor or vegetation, particularly at the side of Entomobryidae and Symphypleona. Their abundance in mature soil is set at 50–a hundred 000 human beings m^−2^ [1]. Mites stay in litter and air-stuffed pores of the soil. Mesostigmata is one of the largest agencies of loose-living mites in soil surroundings [4]. Their density in the soil of wooded areas may be loads of masses per person m^−2^. Oribatid mites, for instance, feeding on plant clutter, are found in an immoderate amount of approximately 25,000–500,000 people m^−2^ [5]. Yet, they continue to be undetected because of their small duration. In addition, the Formicidae dominates in agricultural areas, grasslands, and deserts [6, 7].

RETRACTED

Protura and Diplura are also wingless insects that seem like Collembola. Protura feed on sucking the outer protecting of fungal hyphen and are generally observed in herbal soils. Campodeidae and Japygidae are the two households representing the diplomas. These species are predatory and feed on small fauna. They additionally scavenge on useless natural depend, roots, and so on. Other foremost macroarthropods are dipterans, coleopterans, and hymenopterans consisting of their juveniles. Ants, millipedes, and termites perform the herbal be counted quantity's fragmentation and transportation in deeper soil layers, thereby burrowing inner. So, they appeared as engineers of soil devices. Pauropoda is a whitish millipede-like (>1 mm) species that feed on decaying plants that rely on fungi and carrion. In contrast, some species are predatory. Symphyla is 1–8 mm in duration and determined on the entire natural loam soil feeding on living plant tissues. Tardigrada, Copepods, and terrestrial Isopoda are frequently observed in moist woodland flooring. These species perform the role in the decay of leaf litter and timber residue. Chilopodaare typically predators in soil and litter layers feeding on small arthropods. Millipedes enhance soil devices by coprophagy predominant inside the route of mineralization. Their faces are located with lots of mineral content material. Spiders and pseudoscorpions are predatory arachnids [1].

The arthropod's body is covered with a hard protective coat, and ridges are different in colors and maybe one or mixed. The specialization of body region modifies metamerism for a specific function (stigmatization). The chitinous skeleton gives backing and assurance and is adjusted in tactile structure. The arthropod body is made from an arrangement of the fragment, and each section bears a couple of members. Their body is isolated into the fragmented structure on the outer side, yet inward cavities are not separated like this. Arthropods' exoskeleton comprises fingernail skin, a noncell material emitted by the epidermis of their skin organs [8]. Their fingernail skin shifts in each species, yet for the most part, comprised of three principle layers: the external layers are epicuticle, a dainty, and Waxy coat that dampness confirmations the alternative layer and supply them a few insurances. The exocuticle and endocuticle accommodate chitin and synthetically solidified proteins and unhardened proteins one at a time. Each body portion and appendage area is encased in solidified fingernail skin. The joints between body portions and appendages are secured by adaptable fingernail skin.

The exoskeletons of most oceanic creatures are biomineralized calcium carbonate removed from the water. Some earthbound shellfish created a calcium carbonate exoskeleton, and land creatures cannot depend on a consistent gracefully broken calcium carbonate [9]. Biomineralization typically impacts the exocuticle and the external aspect of the endocuticle [10]. Two speculations about the advancement of biomineralization in arthropods and another pack of creatures delicate that it award relentless guarded reinforcement and permits the creatures to develop in amount and more grounded by giving more inflexible skeletons [11].

RETRACTED

The fingernail skin groups bristle developing from extraordinary cells in the epidermis. Setae (bristle) are as change fit as a fiddle and capacity as limbs. They are utilized as a tangible organ to distinguish air or water flows or product interactions. Amphibian arthropods are used as quills to extend the swimming extremities' surface area and distinguish food particles from water, and sea-going bugs are utilized as air-breathers [12]. Although all arthropods within the exoskeletons muscles are connected to show their appendages, some utilize water-driven strain to pull out. For instance, all creepy crawlies develop. Their legs are solid and can generate pressure up to their resting level often [13]. Their exoskeleton has two layers, epicuticle and procuticle. Ecdysis happens during development. The diversity of the living beings is straightforwardly related to territory, condition, and food accessibility. During this cycle, they produce the specific traits as well as the linkages (both interspecific and intraspecific) that direct the many biological system capacities that are available over the course of a developmental timeline. Soil as territory directs soil arthropod assorted variety dependent on its physical structure (porosity), supplement accessibility, water (soil dampness), state (temperature, pH), and organization of substances [14].

An arthropod plays a key part in keeping up an environment's normal assets and solidness. Predator and parasitoid arthropods offer important support by keeping up horticultural efficiency and decreasing the requirement for agricultural pesticide contributions every year. Other than their utilization in preservation science, they are likewise significant for controlling irritations in agribusiness. Arthropods have interceded environment administrations incorporate yield fertilization and nuisance control [15]. Nearby populace elements affected the dispersal capacity and searching reach. Trophic level impacts the circulation of species.

At the upper surface of the soil, the microarthropod network is a significant part of soil biodiversity and connects with the whole framework segment. An even soil arthropod network is basic in deteriorating crop deposits to frame humus and reusing mineral supplements for progressive harvests [16]. Arthropods add to human food gracefully, legitimately, and significantly more by implication as a pollinator of yields. A few animal types are known to spread extreme malady to human animals and yields. They are the major groups of freshwater, land, air, and marine life, and they are the only two major groups that have adapted to dry environments. The other major group is the amniotes, whose live members are reptiles, birds, and warm-blooded animals [17].

RETRACTED

Evaluations of the number of arthropod species change somewhere between 1,170,000 and 5 to 10 million and account for over 80 percent of all recognized species of living creatures. The number of species stays hard to decide. This is because the evaluation demonstrates presumptions extended to different locales. Hence, an inquiry in 1992 found that in Costa Rica alone, there were 500,000 forms of creatures and plants, of which 365,000 were arthropods [18]. The main objective of this study is to identify the soil arthropods and their level of abundance in the soil of four plant trees, Neem (*Azadiarachta indica*), guava (*Psidium guajava*), mango (*Mangifera indica*), phalsa (*Grewia asiatica*), and their direct association with pH contents, organic, and inorganic contents in soil.

## 2. Material and Methods

### 2.1. Geographically Position of the Experimental Zone

The geographical location of Dera Ghazi Khan is 30′03^″^ N and 70′38^″^ E. The characteristic of climate is dry and little rainfall. The summer is hot, and winter is mild; the average temperature of summer is 42°C, and the winter temperature is 4°C. Windstorms are common in summer due to the barren mountains of koh-suleman and the sandy soil of the area. The highest temperature is present in summer; Fort Munro is on the edge of Punjab and has cooler weather. Scattered snowfall has been reported.

The experiment was performed in the General Zoology Laboratory of Ghazi University of Dera Ghazi Khan to quantify the soil arthropods in urban forests.

### 2.2. Time Duration of the Study

From Nov 2019 to March 2020 was the time duration of study. Samples were taken from four trees, including guava (*Psidium guajava*), mango (*Mangifera indica*), neem (*Azadirachta indica*), and phalsa (*Grewia asiatica*). Samples were collected from three locations: DC Garden D.G. Khan, Mustafa chowk near BISE D.G. Khan, and Shoriya bypass near Canal City. Sampling months were January, February, and March.

### 2.3. Soil Sample

The soil sample was taken from the Dera Ghazi Khan District from three different areas (DC Garden, Mustafa chowk near BISE D.G. Khan, and Shoriya Bypass near Canal City). Soil samples were taken to the Government Agriculture Laboratory of D.G. Khan for further analysis of mineral composition present in the soil [19].

RETRACTED

### 2.4. Sample Collection

The sample for different forest trees in different duration through the Standard Augar. Standard Augar was a 1.5^″^ of diameter and 15^″^ in length with a T-shaped handle. This was subjected to the forest trees where the study was conducted. Samples were collected in three different months, such as Jan, Feb, and March. Samples were taken at three different locations each month [20]. In the form of a triplet, three samples were obtained from each field for 7 days. The total samples for each month are 12, and 36 are total experimental units. The sample was wrapped in plastic bags and taken to the Department of Zoology, Ghazi University Dera Ghazi Khan laboratory, where further sample evaluation was carried out (Figure 1).

### 2.5. Apparatus

Apparatus used for the collection of samples and identification of collecting species were burlesque funnel, beaker, flask, microscopic slides, and liquid measurement glass.

### 2.6. Extraction of Arthropods

The samples were extracted through the burlesque funnel method. The sample of soils was kept in the funnel on guaz/filter paper having diminutive minuscule apertures, which sanction to pass these arthropods from apertures due to heat and light fitted at the top of the funnel. After putting soil in the funnel, we utilized light to engender heat and kept this heat light on the soil for one week. We reiterate this method with every sample of soils amassed from different plant trees and sites [21]. Beneath the funnel, a solution of ethanol (30%) and distilled water (70%) keeping, and due to the heat and light of the bulb, minuscule arthropods will move in the antithesis direction of light and heat. These arthropods will move forward to that solution which is kept beneath the funnel (Figure 2).

### 2.7. Chemical and Reagents

#### 2.7.1. Solution

The solution is prepared, which consists of ethanol (30%) and distilled water (70%). Soil samples were put into a funnel, provision the light of a 100-watt bulb because arthropods are heat sensitive. Therefore, arthropods move towards the bottom. The solution can attract the soil arthropods [22].

### 2.8. Soil Samples Analyses

To determine the different components of soil samples, some analyses were performed in the soil testing laboratory of the agriculture department of D.G. Khan.

#### 2.8.1. Chemical Analyses of Soil Samples from Different Tree Plants

To study the nature of the soil in terms of organic matter, pH, moisture content, electric conductivity phosphates (PO_4_), and potassium (K) according to standard methods for soil analysis. The moisture content of soil samples was also determined. Details of soil sample analyses are described as follows.

RETRACTED

#### 2.8.2. pH

The pH of samples was determined in the laboratory using a “Digital pH meter (D-25 Horiba)”.

#### 2.8.3. Electrical Conductivity (E.C)

The EC of soil samples was determined with the help of “Conductivity meter model WTWcind330i.”

#### 2.8.4. Phosphates

The 4500-P standard method was used to determine the sample's level of phosphates (APHA, 2005).

#### 2.8.5. Potassium

Soil potassium extraction with ammonium-acetate (NH_4_OAc) from oven-dried samples was used to determine potassium. To determine the potassium content of the filtered extracted, we can use Jenway PFP7 Flame Photometer.

#### 2.8.6. Moisture Content

The moisture content of the soil was determined using a simple Memmert incubator (oven) (Model INB 300).

### 2.9. Identification of Arthropods

The arrangement with the arthropods was moved for the minute investigation to distinguish the arthropods and gauge the insects' thickness. The identification of the insects was accomplished by using a stereoscope (Bresser GmbH's Science ETD-201, Art No. 58-06200, Lot No. 5806200-1617) in conjunction with a high-definition camera and a personal computer screen, both of which were located in the laboratory of the Zoology Department at Ghazi College in Dera Ghazi Khan (Figure 3). We took photographs of various soil arthropods available in this isopropyl arrangement. The arrangement was put onto the slides, and with a high-goal camera associated with a stereoscope and screen, we took the photographs of various soil arthropods and spared them in PC. Later, ID was finished [23].

### 2.10. Diversity Analyses

Some of the following diversity indices were employed to calculate the diversity in observed soil arthropods: *T*-test, Shannon Weiner, cluster analysis, species abundance, species richness and similarity index, evenness, dominance, and maximum diversity.

#### 2.10.1. Species Richness

The presence of species in a specific region was calculated with the help of samples.

#### 2.10.2. Species Diversity

The accumulation of a different type of species in a given community was calculated.

#### 2.10.3. Relative Species Abundance

The proportion of any specific species as compared to other species was measured. The percentage of any particular species compared to the total species in the area was also measured.

#### 2.10.4. Dominance

The dominance of arthropods was studied by calculating the relative abundance of arthropods identified from each soil sample. The species is present in more numbers than other species in a given community.

RETRACTED

#### 2.10.5. Evenness, Species Abundance, and Diversity Index

To compare the similarity of all species in a given population. The number of individuals per species was calculated. The diversity index was used to calculate the species in a given community.

### 2.11. Statistical Analysis

*T*-test was used to analyze the *p* values.

Shannon index was used to find out the species diversity in the sample.

Shannon Index (*H*) = −∑*p*_*i*_ ln *p*_*i*_*i* = 1.

Shannon index tells us about the diversity of species in the sample.

*p* is the proportion of particular species in the total number of individual species, *n*/*N* is the no. of species in the natural log, and *Σ* is the sum of the calculations.

## 3. Results

### 3.1. Soil Sample Analysis Report

In this study, we have discussed the findings of our experiment. The experiment was laid out to check the biodiversity of arthropods in different soil samples under different types of trees, i.e., *Psidium guajava*, *Azadirachta indica*, *Grewia asiatica*, and *Mangifera indica*. The discussion of the findings of the results is given below (Table 1).

### 3.2. Estimation of Arthropods in Neem (*Azadirachta indica)*

There were total 12 numbers of species of arthropods that were found in the soil. The maximum number of species found in *Azadirachta indica* during January was mites (50), followed by millipedes (41) and centipedes (40). The minimum number of arthropods found in the soil was termites (8). During February, the maximum number of species found was mites (51), followed by springtail and ants (47) and millipedes (43), while the minimum numbers of arthropods were wolf spider, which was counted at 21 in February. During March, the maximum number of species of arthropods was a centipede, and ants counted 54, followed by mites, 53, and millipede, 48, while the minimum number of species was a wolf spider, 30. The maximum number of 12 species of arthropods was highest in March 535, followed by February 453 and January 361. (Table 2).

### 3.3. Relative Abundance of Arthropods in *Azadirachta indica*

Relative abundance % during January and February was found to be highest for mites, and during March, it was found to be highest for ants, springtail, and centipedes.

### 3.4. Estimation of Arthropods in *Psidium guajava*

There were a total of 12 numbers of species of arthropods that were found in the soil. The maximum number of species found in *Psidium guajava* during January was centipedes (39), followed by ants (37) and millipedes, springtail, and oribatid mites (36). The minimum number of arthropods found in the soil was termites (16). During February, the maximum number of species found were centipedes (49), followed by ants (46) and millipedes (43), while the minimum number of arthropods was termites, which were counted at 25 in February. During March, the maximum number of species of arthropods were ants counted at 55, followed by millipedes and centipedes, 54, while the minimum number of species were wolf spiders at 29. The maximum number of a total of 12 species of arthropods was found highest during March 518, followed by February 440 and January 356. (Table 3).

RETRACTED

### 3.5. Relative Abundance of Arthropods in *Psidium guajava*

Relative abundance % during January and February was found to be highest for centipedes, and during March, it was highest for ants.

### 3.6. Estimation of Arthropods in *Mangifera indica*

There were total 12 numbers of species of arthropods that were found in the soil. The maximum number of species found in Mangifera indica during January was millipedes, centipedes, mites, and springtail (32), while the minimum number of arthropods found was termites (18). During February, the maximum number of species found was mites (42), followed by ants and oribatid mites (39). The minimum number of arthropods was a pseudoscorpion, and wolf spider counted 23 each in February. During March, the maximum number of species of arthropods was mites, springtail, and ants counted at 50, while the minimum number of species was wolf spider 22. The maximum number of a total of 12 species of arthropods was found highest during March 494, followed by February 390 and January 325 (Table 4).

### 3.7. Estimation of Arthropods in *Grewia asiatica*

There were total 12 numbers of species of arthropods that were found in the soil. The maximum number of species found in Grewia asiatica during January was mites (33), while the minimum number of arthropods found was termites (14). During February, the maximum number of species found were ants (46), followed by springtail (44), while the minimum number of arthropods was oribatid mites, which were counted 14 in February. During March, the maximum number of species of arthropods was centipedes that counted 61, while the minimum number of species was oribatid mites, 16. A maximum number of total of 12 species of arthropods was found highest during March 531, followed by February 416 and January 332 (Tables 5 and 6).

### 3.8. Shannon-Weiner Index

The Shannon diversity index measured the difference in the diversity of trees.  Table 7 below presents the diversity indices of arthropods among selected tree species i.e., *Azadirachta indica*, *Mangifera indica*, *Grewia asiatica*, and *Psidium guajava*. Accordingly, the diversity of arthropods was significantly different among all selected tree species. The highest diversity was observed in samples 1 of Mangifera indica and 3 of Azadirachta indica (*H*′ = 2.47) followed by samples 2 and 3 of *Psidium guajava* and *Mangifera indica* (*H*′ = 2.46).

RETRACTED

### 3.9. Cluster Analysis

In this dendrogram, it is evident that in *Psidium guajava* and *Grewia asiatica*, population of millipede is more similar to other trees. *Mangifera indica* has the highest number of millipedes and is more different than any other tree. Similarly, the population of sow bugs in *Azadirachta indica* and *Grewia asiatica* is similar, and Psidium guajava and Mangifera indica are similar. Still, the highest number of sow bugs was found in the *Grewia asiatica* and *Psidium guajava*. Cluster analysis showed that the number of spiders in *Azadirachta indica* and *Psidium guajava* was similar, while the highest number of spiders was found in *Mangifera indica*. As far as the pseudoscorpion is concerned, cluster analysis showed that Mangifera indica and Grewia asiatica have similar numbers. In contrast, *Psidium guajava* and *Azadirachta indica* have a similar number of pseudoscorpions, while the highest number of pseudoscorpions was found in the soil taken from *Psidium guajava* and *Mangifera indica* (Figure 4).

Cluster analysis for wolf spiders showed that *Psidium guajava* and *Mangifera indica* have a similar number, and *Azadirachta indica* and *Grewia asiatica* have the same number of wolf spiders. It can be seen from the graphs that *Grewia asiatica* and *Psidium guajava* had the highest number of wolf spiders. For centipedes, it is evident that *Azadirachta indica* and *Psidium guajava* had a similar number of centipedes, while the maximum number of centipedes was present in *Grewia asiatica* as compared in the cluster analysis. The maximum number of mites was present in the soil taken from the *Psidium guajava* and *Mangifera indica*. In contrast, the maximum number of tiger beetles was also present in the same tree species as in mites (Figure 5).

There was less or no difference in the presence of spider tail numbers in *Mangifera indica* and *Azadirachta indica*. In contrast, the maximum number of spider tails were present in *Psidium guajava*. As far as oribatid mites are concerned, the maximum number of these arthropods was present in *Psidium guajava* and *Mangifera indica*. The maximum number of termites and ants was also present in *Psidium guajava,* as indicated by the cluster analysis dendrograms (Figure 6).

### 3.10. Arthropod Diversity

The graph below represents the total number of arthropods in the sample collected in the experiment. The results are given in the number of each arthropod species and the percentage. The total number of arthropods in the experiment was 5151, millipedes contributed 10% (499) of the total population, and the sow bug represented 7% of the total population which was 353. The number of spiders accounted for 9% (468), the number of pseudoscorpions accounted for around 7% (357), and the number of wolf spiders accounted for 7% (349). There were 528 centipedes (ten percent), but there was only a difference of two mites (526, ten percent). Tiger beetles were found in 365 (7%) of the overall population, springtails numbered 522 (10%), and oribatid mites made up 7% (372) of the whole population (Figure 7). In the samples taken for the trials, the number of termites was the lowest, contributing just 6%, and there were only 285. In contrast, the percentage of ants was 10%, with 522 of them (Table 8).

RETRACTED

## 4. Discussion

For the analysis of the soil characteristics, samples from the experiment sites were taken and sent for analysis. The analysis report is given in Table 1. It is evident from the report that the soil was normal and needed no amendments, i.e., the addition of gypsum etc., to overcome the problem of salts depletion or salt deposition on the surface of the soil. From the results, it is concluded that EC of the soil lies in between 2.94 and 4.92 ms/cm. Soil pH in Pakistan fall in very optimum range so as our sample does, pH of the samples fall in the range of 7.02–7.58. Organic matter in the soil is the main characteristic that defines the fertility of the soil. The maximum organic matter % of the sampled soil was 0.92, and the minimum % was 0.42. Available phosphorus and potassium of the soil lies in between 7.32 and 8.42 and 176 and 196, respectively. Saturation % of the sampled soil was the same for the entire sample, 36, while the soil texture was loam, according to the soil analysis report.

In our study, more arthropods are captured compared to those that report arthropods in the agronomic crops. According to previous studies, the near-natural habitat offers arable land, stable protection, a food source, and a microclimate for various arthropods [23]. Therefore, more arthropods can be caught near the orchard.

For a long time, people have believed that plant diversity is an important factor in determining nutrient-rich biodiversity [24]. The close relationship between the composition of plants and arthropods is complex and beyond the scope of this study. However, this study has shown that “habitat complexity” significantly impacts the abundant arthropods in the soil. Therefore, our results agree with those of [25] observed that the frequency of arthropods generally decreases with increasing land use and management intensity. These authors believe that the entire process of agriculture intensification, from full local vegetation associations to fragmented mixed agricultural landscapes to high-intensity farming or pasture systems, can create a range of impacts and threats that lead to biodiversity reduce. Many possible explanations exist for the abundance of arthropods in less land-intensive systems [26]. Areas with little to moderate improvement/intensification (such as indigenous vegetation and pastures) may have greater habitat complexity because the risk of intensification and uniform management is lower than that of many agricultural systems. Therefore, there can be many niche opportunities with complex land use, while fewer niches are available for systems with less complex structure and composition. Therefore, in a simplified system, the possibility of coexistence by resource allocation can be reduced, reducing species abundance.

RETRACTED

The habitat's more complex composition and structure may offer humans more opportunities to obtain a wider range of alternative food resources [27], which helps classify omnivorous and nonspecific predatory organisms. Another possible explanation for the increase in wealth in less disturbed habitats is that in environments with frequent or severe disturbance, the composition of the community cannot go beyond the initial pioneering stage. Frequent “resetting of the continuous clock” in areas of high disturbance results in an environment conducive to the first continuous species but not to the later continuous species [28]. If the disorder is severe and common (e.g., in intensive farming), all but the most diverse group can be excluded, reducing the total number of species.

Soil arthropods react differently to light. One explanation is that light can speed up the sample drying rate to reflect it compared to extraction without light. On the contrary, soil arthropods are more sensitive to an increase in temperature or a decrease in humidity. In this case, the use of light during the extraction process inactivates the arthropod before exiting the sample, so its apparent abundance decreases. In addition, soil arthropods live in relatively cool and dark (soil) habitats [14]. They can therefore react sensitively to increased temperature and incidence of light, so that the use of light in the extraction process can lead to an underestimation of soil arthropods. The immature soft epidermis makes it more susceptible to moisture droplets in the suction cup. Organisms such as mites (the vast majority of young animals in this study) are inactive during moulting and, therefore, cannot leave the sample [29]. As a result, another extraction method, such as flotation, should be more suitable for the immature form.

RETRACTED

In March, soil arthropods left the sample faster. Similarly, the March samples had the highest frequency, while the January samples had the low frequency. One explanation is that the loose structure of the sample stores less moisture and dries faster, so the temperature/moisture gradient can be established more quickly than with compact samples, which can store more moisture [30].

This has a double effect: over a month, the gradient created by drying the sample at room temperature slowly moves down, forcing the arthropods to leave the sample, but their size is not large enough to kill them, translating into a greater abundance of arthropods. In March, the gradient created by drying the sample at room temperature reached a higher critical level. It became larger, forcing the arthropods to move outward, resulting in a higher estimate of the frequency of arthropods in the sample. This can also be elaborated by the fact that during January the richness of the soil in terms of fertility or organic matter is enhanced during March due to moderate temperature and humidity.

Compared to traditional methods, organic farming can also increase the abundance of many species and biota. For example, the use of herbicides in conventional agricultural systems will reduce the incidence of weeds in nature. Depending on the species of these plants, this can have harmful effects on insects and birds [31]. Similarly, the use of insecticides will reduce not only pests but also predatory insects.

Common methods of plant management such as deep ploughing, the application of agrochemicals, and mechanical harvesting can increase the frequency and severity of interference systems [32]. We have not analyzed the effects of these factors in our research. However, we are studying agricultural and nonagricultural systems [33] which showed that agriculture in the vineyard system destroyed the numbers of invertebrates, including ants, pennies, and millipedes. Agriculture in particular destroys the combination of ants [34] which found a similar conclusion in the olive tree ecosystem: if olive trees are frequently disturbed, sensitive ant species are gradually eliminated.

Many arthropods now become serious pests due to excessive use of pesticides without any proper recommendations on all types of fruit plants especially. These pesticides may also cause the reduction of arthropods which are the common source of soil reclamation by decomposing with the help of bacteria in their bodies. Mango, guava, and falsa trees are susceptible to various insects and mites. It is known that there are 400 pests on these trees reported in different parts of the world [35]. According to the precise classification of the infestation parts of the pests, the main (about 45% of total species) is branch and leaf food, followed by fruit food (32%), and the rest feed on inflorescences, branches, and trunks. Secondary pests can become serious due to cultural customs or climatic and/or species changes or the indiscriminate use of pesticides on the main pests. [36] reported that large-scale insects became serious pests due to the ruthless use of insecticides on fruit flies. Similarly, mites, considered minor pests, can become serious due to human interference. Occasional or sporadic pests can cause economic losses in local areas even at a specific time.

RETRACTED

Our results suggest that agricultural orchards affect soil arthropods in all areas. Arthropods are important drivers of ecosystem functions as nutrient cycling, pest control, pollination, and maintenance of soil structure. So, strategies for addressing the conservation of arthropods in agricultural orchards must be promoted.

## 5. Conclusion

Different kinds of trees were selected to check the diversity of arthropods. The total number of arthropods in the experiment was 5151, in millipedes 10%, spiders accounted for 9%, sow bug, pseudoscorpion, wolf spider, and tiger beetles were present in 7% of the total population. *T*-test and statistical analysis showed that the results were significant. The Shannon diversity index of the arthropods is also developed. Similarly, the highest dissimilarity in the number of sow bugs was found in the phalsa and guava, for spiders in mango, pseudoscorpion and mites in guava and mango, centipedes in phalsa, oribatid mites, and for termites, ants and spider tails were present in guava.

## Figures and Tables

**Figure 1:** Standard Augar used for the sampling procedure during field survey.

**Figure 2:** Installation of berlese funnels to extract insects from soil samples. It uses a heat source (in this case, a light bulb) to dry the sample, forcing the insects through a screen and into a jar of preserving fluid.

**Figure 3:** Stereoscope was used to visualize the respective arthropods for their examination during this study.

**Figure 4:** Cluster analysis of millipedes, sow bug, spider, and pseudoscorpion species in all observed trees to construct groups, or clusters, while ensuring that within a group, the observations are as similar as possible. In contrast, observations belonging to different groups are as different as possible.

**Figure 5:** Cluster analysis of wolf spider, centipede, mites, and tiger beetle species in all observed trees to construct groups, or clusters, while ensuring that within a group, the observations are as similar as possible, while observations belonging to different groups are as different as possible.

RETRACTED

**Figure 6:** Cluster analysis of spider tail, oribatid mites, termites, and ants species in all observed trees to construct groups, or clusters, while ensuring that within a group, the observations are as similar as possible. In contrast, observations belonging to different groups are as different as possible.

**Figure 7:** Arthropod diversity in the sampled tree soil during January, February, and March.The diversity has been shown in terms of numbers as well as percentage.

**Table 1:** Soil analysis was done for the different sites of experimental areas. For this purpose, several soil parameters (EC, pH, organic matter percentage, available P and K, soil saturation, and texture) were considered.

Parameter	Soil sample sites											
	DC Garden				Mustafa Chowk				Canal City			
ECe (ms/cm)	Neem	Guava	Mango	Phalsa	Neem	Guava	Mango	Phalsa	Neem	Guava	Mango	Phalsa
	1.88	1.71	4.85	3.12	1.56	1.98	4.92	2.94	1.6	1.75	4.32	3.23
Soil pH	7.61	7.59	7.52	7.02	7.65	7.78	7.58	7.28	7.69	7.58	7.32	7.33
Organic matter (%)	0.79	0.66	0.88	0.56	0.66	0.77	0.92	0.42	0.72	0.62	0.77	0.67
Available phosphorous (ppm)	8.26	7.67	8.32	7.92	7.72	8.72	8.42	7.96	8.56	8.52	8.18	7.32
Available potassium (ppm)	226	182	186	182	195	195	196	184	190	175	192	176
Saturation (%)	38	38	36	36	38	38	36	36	38	38	36	36
Texture	Loam	Loam	Loam	Loam	Loam	Loam	Loam	Loam	Loam	Loam	Loam	Loam
Remarks	Normal soil	Normal soil	Normal soil	Normal soil	Normal soil	Normal soil	Normal soil	Normal soil	Normal soil	Normal soil	Normal soil	Normal soil

**Table 2:** The total numbers of arthropods in *Azadirachta indica* were counted during all three sampling months.

Arthropods species	*Azadirachta indica* (Jan)	*Azadirachta indica* (Feb)	*Azadirachta indica* (March)
Millipedes	41	43	48
Sow bug	21	32	36
Spider	34	42	47
Pseudoscorpion	27	32	34
Wolf spiders	16	21	30
Centipedes	40	42	54
Mites	50	51	53
Tiger beetle	26	38	43
Springtail	37	47	54
Oribatid mites	22	37	47
Termites	8	21	35
Ants	39	47	54
	361	453	535

**Table 3:** The total numbers of arthropods in *Psidium guajava* were counted during all three sampling months.

Arthropods species	*Psidium guajava* (Jan)	*Psidium guajava* (Feb)	*Psidium guajava* (March)
Millipedes	36	43	54
Sow bug	17	29	38
Spider	34	41	45
Pseudoscorpion	29	30	31
Wolf spiders	29	35	29
Centipedes	39	49	54
Mites	29	40	50
Tiger beetle	18	34	41
Springtail	36	42	52
Oribatid mites	36	26	35
Termites	16	25	34
Ants	37	46	55
Total	356	440	518

RETRACTED

**Table 4:** The total numbers of arthropods in *Mangifera indica* were counted during all three sampling months.

Arthropods species	*Mangifera indica* (Jan)	*Mangifera indica* (Feb)	*Mangifera indica* (March)
Millipedes	32	34	47
Sow bug	24	29	39
Spider	28	38	43
Pseudoscorpion	26	23	30
Wolf spiders	20	23	22
Centipedes	32	37	49
Mites	32	42	50
Tiger beetle	24	24	34
Springtail	32	38	50
Oribatid mites	28	39	46
Termites	18	24	34
Ants	29	39	50
Total	325	390	494

**Table 5:** The total numbers of arthropods in *Grewia asiatica* were counted during all three sampling months.

	*Grewia asiatica* (Jan)	*Grewia asiatica* (Feb)	*Grewia asiatica* (March)
Millipedes	29	41	51
Sow bug	19	31	38
Spider	28	39	49
Pseudoscorpion	31	29	35
Wolf spiders	32	38	54
Centipedes	29	42	61
Mites	33	42	54
Tiger beetle	30	25	28
Springtail	31	44	59
Oribatid mites	26	14	16
Termites	14	25	31
Ants	30	46	55
	332	416	531

**Table 6:** Statistical analyses of all four respective tree samples were done. Three samples from each tree were taken under consideration. Following results showed that the entire samples have a significant level of arthropods.

Name and sample	*T* test	*p* value
*Azadirachta indica* 1	8.60	0.000^∗∗∗^
*Azadirachta indica* 2	13.46	0.000^∗∗∗^
*Azadirachta indica* 3	17.54	0.000^∗∗∗^
*Psidium guajava* 1	12.33	0.000^∗∗∗^
*Psidium guajava* 2	15.91	0.000^∗∗∗^
*Psidium guajava* 3	15.43	0.000^∗∗∗^
*Mangifera indica* 1	19.49	0.000^∗∗∗^
*Mangifera indica* 2	15.31	0.000^∗∗∗^
*Mangifera indica* 3	15.30	0.000^∗∗∗^
*Grewia asiatica* 1	17.02	0.000^∗∗∗^
*Grewia asiatica* 2	12.28	0.000^∗∗∗^
*Grewia asiatica* 3	10.76	0.000^∗∗∗^

**Table 7:** Shannon-Wiener index (Shannon-Weiner index) describes the disorder and uncertainty of individual species. Higher uncertainty means the higher the diversity.

Trees	No. of species	Sample 1 (*H*′)	No. of species	Sample 2 (*H*′)	No. of species	Sample 3 (*H*′)
*Azadirachta indica*	361	2.40	416	2.45	535	2.47
*Psidium guajava*	356	2.45	390	2.46	518	2.46
*Mangifera indica*	325	2.47	440	2.46	494	2.46
*Grewia asiatica*	332	2.46	453	2.44	531	2.43

**Table 8:** Total numbers of arthropod species found in all experimental sites on four respective trees.

Arthropods species	Experimental sites												
	DC Garden				Mustafa Chowk				Canal City				
	Neem	Guava	Mango	Phalsa	Neem	Guava	Mango	Phalsa	Neem	Guava	Mango	Phalsa	Total
Millipedes	41	36	32	29	43	43	34	41	48	54	47	51	499
Sow bug	21	17	24	19	32	29	29	31	36	38	39	38	353
Spiders	34	34	28	28	42	41	38	39	47	45	43	49	468
Pseudoscorpion	27	29	26	31	32	30	23	29	34	31	30	35	357
Wolf spiders	16	29	20	32	21	35	23	38	30	29	22	54	349
Centipedes	40	39	32	29	42	49	37	42	54	54	49	61	528
Mites	50	29	32	33	51	40	42	42	53	50	50	54	526
Tiger beetle	26	18	24	30	38	34	24	25	43	41	34	28	365
Springtails	37	36	32	31	47	42	38	44	54	52	50	59	522
Oribatid mites	22	36	28	26	37	26	39	14	47	35	46	16	372
Termites	08	16	18	14	21	25	24	25	35	34	34	31	285
Ants	39	37	29	30	47	46	39	46	54	55	50	55	527

RETRACTED

## Data Availability

All data relevant to this paper will be available to readers upon request from the corresponding authors.
